# Deep Learning-Based Chest CT Image Features in Diagnosis of Lung Cancer

This article has been retracted.

**DOI:** 10.1155/2022/4153211

**Published:** 2022-01-19

**Authors:** Jianxin Feng, Jun Jiang

**Affiliations:** Department of Interventional Therapy, People's Hospital of Baoji, Baoji City, 721000 Shaanxi Province, China

## Abstract

This study was to evaluate the diagnostic value of deep learning-optimized chest CT in the patients with lung cancer. 90 patients who were diagnosed with lung cancer by surgery or puncture in hospital were selected as the research subjects. The Mask Region Convolutional Neural Network (Mask-RCNN) model was a typical end-to-end image segmentation model, and Dual Path Network (DPN) was used in nodule detection. The results showed that the accuracy of DPN algorithm model in detecting lung lesions in lung cancer patients was 88.74%, the accuracy of CT diagnosis of lung cancer was 88.37%, the sensitivity was 82.91%, and the specificity was 87.43%. Deep learning-based CT examination combined with serum tumor detection, factoring into Neurospecific enolase (N S E), cytokeratin 19 fragment (CYFRA21), Carcinoembryonic antigen (CEA), and squamous cell carcinoma (SCC) antigen, improved the accuracy to 97.94%, the sensitivity to 98.12%, and the specificity to 100%, all showing significant differences (*P* < 0.05). In conclusion, this study provides a scientific basis for improving the diagnostic efficiency of CT imaging in lung cancer and theoretical support for subsequent lung cancer diagnosis and treatment.

## 1. Introduction

With the witness of the rapid development of economy, culture, and technology in Chinese society, every Chinese has a genuine sense of joy. However, social development usually occurs with the change of human living environment, which results in the changes in the occurrence of different diseases to some extent. The impact of the changes in the incidence of lung diseases is the most significant. The incidence of multiple lung disease is enhanced, especially lung cancer [1–3]. Among that of various cancer diseases, the incidence and mortality of lung cancer are both at high levels with the rapidly growing trend year by year. In 2018, its growth rate was about 27% with a rising trend [4]. At early phase, lung cancer is imperceptible because of no other specific clinical manifestations. The main manifestation of early lung cancer is pulmonary nodules, which can be detected by other examinations. Some significant symptoms (fever, hemoptysis, and short breath) reveal that patients suffer from the diseases at middle or advanced phases. For these patients, the optimal treatment time is missed with poor prognosis [5, 6]. Therefore, early diagnosis and early treatment are of great significance in the prognosis of lung cancer patients.

At present, the main examination method of lung diseases is imaging detection mainly by computed tomography (CT) [7]. CT technology is based on X-ray and widely applied in clinical practice. Besides, it plays an essential role in the examination and diagnosis of lung diseases, especially in the examination of lung functions. However, CT shows the disadvantage in the diagnosis methods of diseases, which is the impacts of subjective factors on the results of film review by doctors. Furthermore, diagnosis results are affected to some extent [8]. The major observation points and thinking modes of doctors with different work experience are both different in reviewing the same CT image. Consequently, there are usually differences in the results. Besides, the surge in the number of patients in contemporary society also cause the increase in the pressure of film review on doctors.

Radiologists have now determined some of the visual physical characteristics, such as lesion size, attenuation, assessment, and surrounding cystic airspace, to distinguish from benign or malignant lesions. The radiological characteristics can quantitatively capture the shape, size, volume, and texture of the tumor or normal tissue area. They can be combined with artificial intelligence to form a prediction model of prognosis [9, 10].

At present, there are challenges faced by chest CT scans for cancer diagnosis in two aspects. First, a system must be developed for chest CT diagnosis to accurately extract phenotypic features from images. Second, the system must identify which phenotypic characteristics are related to the underlying genotype and disease behavior among thousands of phenotypes, to provide further help for the prognosis and clinical treatment of the disease [11]. Mask Region Convolutional Neural Network (Mask-RCNN) algorithm model is based on Faster-Regions with Convolutional Neural Network (Faster-RCNN) and combines detection and classification. Studies have shown that Mask-RCNN is the most advanced deep learning model and has good application effects in dynamic video detection and segmentation [12]. Other studies have proposed that the automatic segmentation effect of Mask-RCNN algorithm is conducive to the classification and recognition of diseases [13]. Dual Path Network (DPN) is a CNN, which combines the advantages of aggregation residual transform (ResNeXt) for feature reuse and dense convolutional network (DenseNet) for exploring new features [14], and has a good application effect in the automatic detection of pulmonary nodules.

To conclude, the automatic segmentation model of optimization-based Mask-RCNN algorithm was adopted to process CT detection images of lung cancer and examine lung functions of lung cancer patients. Besides, serum tumor detection was utilized to assess its identification effects on benign and malignant tumors. The adoption and assessment of the model provided scientific and reasonable research basis for improving clinical diagnosis and treatment levels of lung cancer patients.

## 2. Materials and Methods

### 2.1. Research Subjects

In this study, 45 patients diagnosed with lung cancer by surgery or puncture in hospital in a certain area were selected as the observation group. During the same period, 45 patients with benign lung lesions were defined as the control group. All patients had CT and MRI scans and serum tumor marker detection, with complete clinical diagnosis records and imaging data. Of the 90 patients, 54 were male patients, and 36 were female patients. Patients' age ranged between 32 and 79 with the average of 57.23 ± 12.99. The range of lesion diameters was 1.12 to 2.82 cm, and the average diameter was 2.01 ± 0.41 cm. The study had been approved by ethics committee of hospital. The patients and their families had a full understanding of the content and methods of the research and had signed the relevant informed consents.

The patients were included in the research based on the following standards. All patients were diagnosed with lung cancer based on the diagnosis standard for lung cancer; patients did not receive any treatment before the examination; patients had signed the informed consent forms; patients showed normal mental state and consciousness; patients were not allergic to contrast agents; the patients were excluded from the research based on the following standards; patients' CT detection images were incomplete; patients did not experience complete examination and research.

### 2.2. CT Examination

In the research, 16-layer spiral CT scanner was adopted as the examination instrument. The scanning method was whole-body low-dose CT scanning. The scanning parameters included voltage 110 kV, current 90 mAs, thickness 7 mm, layer spacing, and reconstruction interval were 0.9 mm, pitch 0.801, and collimation 15 × 0.8. The scanning process was as follows. Patients took supine position and placed two relaxed arms on two sides. The nodule with the largest number of layers was dynamically enhanced, and then, the range was narrowed. After that, 89 mL of contrast agent was injected (the rate was 4.0 mL/s, and the injected contrast agent was ioversol (320 mgL/mL)).

### 2.3. Serum Tumor Marker Detection

2 mL of fasting venous blood was drawn in the morning for detection and anticoagulated with heparin. Then, it was centrifuged for 10 min at 3000 r/min, and the serum was separated to test. Roche electrochemiluminescence analyzer and supporting kits were used to detect neurospecificity enolase (NSE), cytokeratin 19 fragment (CYFRA21), carcinoembryonic antigen (CEA), and squamous cell carcinoma antigen (SCC), and the operation was carried out in strict accordance with the instructions or relevant operating procedures. Positive standards are as follows: NSE > 16.3 ng/mL, CYFRA21 − 1 > 3.30 ng/mL, CEA > 5.0 ng/mL, and SCC > 1.50 ng/mL.

### 2.4. CT Image Segmentation Based on Mask-RCNN Algorithm Model

The Mask-RCNN algorithm model is based on the Faster-RCNN algorithm, and it is a convolutional neural network model that can be used for both the object detection and image segmentation [15]. Combining target detection and segmentation algorithms, it can efficiently segment the CT image. Unlike the Faster-RCNN algorithm, the Mask-RCNN algorithm replaces the original region of interest (ROI) pooling layer with a better ROI Alignment layer to improve the accuracy of the image in segmenting the boundary [16]. On the basis of the new network model, it uses a full convolutional network for image segmentation, and its structure is shown in Figure 1.

The replacement with the ROI Alignment layer realizes the mutual correspondence between output pixels and input pixels and effectively retains the spatial data contained in the image. In the process, the target pixel position in the original CT image can be calculated by the following equations.

(1) $$\begin{array}{c} SrcW=dstW*\left(\frac{src\text{Width}}{dst\text{Width}}\right), \end{array}$$

(2) $$\begin{array}{c} SrcH=dstH*\left(\frac{src\text{Heigth}}{dst\text{Heigth}}\right). \end{array}$$

In equations (1) and (2), *dstW* and *dstH* refer to the pixel coordinates of area suggestion boxes, *srcW* and *srcH* represent the target pixel coordinates in the original images, *src*Width denotes the width of original images, *src*Heigth means the height of original images, *dst*Width stands for the width of area suggestion boxes, and *dst*Heigth refers to the height of area suggestion boxes.

Bilinear interpolation method was utilized to calculate the pixel value of each unit sampling point, and the maximum pool calculation was carried out, which is shown in equation (3) below.

(3) $$\begin{array}{c} \begin{array}{c} t\left(e+q,g+h\right)=\left(1-q\right)\left(1-h\right)t\left(e,g\right)+\left(1-q\right)ht\\ \left(e,g+1\right)+q\left(1-h\right)+\left(e+1,g\right)+qht\left(e+1,g+1\right). \end{array} \end{array}$$

Equation (3) contains four coordinate points to interpolate in the *M* and *N* directions.

In this study, the loss function is used to train the model, which includes the bounding box regression loss and the target classification loss. The overall loss function is expressed as follows.

(4) $$\begin{array}{c} K=k_{cls}+k_{\text{box}}+k_{\text{mask}}. \end{array}$$

In equation (4), *k*_mask_ refers to mean binary cross entropy loss.

(5) $$\begin{array}{c} \text{Crossentropy}\left(t,0\right)=-\left(t,\log\left(v\right)+\left(1-t\right)\log\left(1-v\right)\right). \end{array}$$

In equation (5), *t* denotes target images, and *v* refers to output results.

Here, different types of targets generate masks of different types of attributes to avoid mutual influence between those of the same type.

### 2.5. CT Detection Based on Three-Dimensional DPN

In addition to using the Mask-RCNN full convolutional network to segment CT images of the lung, three-dimensional DPN based on deep learning can also be used to extract and detect lung lesions, because it is noted that DPN has good performance on ImageNet. Therefore, after comparison, this article chooses the DPN algorithm structure to detect lung lesions in patients with lung cancer. The DPN algorithm has a tightly connected structure like the DenseNet algorithm and applies the residual learning like the ResNet algorithm, so DPN can perform cross-layer learning and achieve effective feature reuse when applying residual learning. At the same time, it can also reduce the use of redundant parameters through a special structure. In the study, the dual-link structure divides the target image map into two parts, as shown in Figure 2. The dual-link link is expressed as follows.

(6) z=Relux:j,Fx:j,Fxj:.xh:,

where *j* is used to describe the ratio of the two parts in the dual-link structure, *z* is the output image map in the structure, and *F* represents the convolutional layer.

### 2.6. Statistical Methods

The SPSS19.0 statistical software was used for data processing. Measurement data was expressed by mean ± standard deviation ($\dot{\text{x}}\pm s$). Count data was expressed as a percentage (%), and *χ*2 test was adopted. *P* < 0.05 indicated significant differences.

## 3. Results

### 3.1. Image Segmentation Results Based on Mask-RCNN Algorithm Model

In the research, highly flexible and portable TensorFlow framework was adopted to establish Mask-RCNN algorithm model. CT examination images of the research objects were utilized as the image data on training. Besides, stochastic gradient descent (SGD) training network was utilized in training with iteration times (epoch), momentum, learning rate, batch size, and weight decay being 400, 0.78, 0.000098, 3.5, and 0.000098, respectively. The results showed that loss function converged after 360 iterations. According to the results, the 400 iteration model was adopted to segment CT images, and the segmentation effects are demonstrated in Figure 3.

In Figure 3, the red box referred to the marker of the position of pulmonary parenchyma by Mask-RCNN algorithm, and the yellow dotted lines represented the automatic segmentation of pulmonary parenchyma by Mask-RCNN algorithm. Based on the above results, Mask-RCNN algorithm could be adopted to segment pulmonary parenchyma. Nevertheless, there were slight errors at boundaries, which suggested that Mask-CNN algorithm could not identify the boundaries of images accurately, but it could segment CT images.

### 3.2. Comparison of Results of Lung Lesion Detection Algorithms Based on Three-Dimensional DPN

CT image data utilized in the research were all the medical image data on the selected subjects. Each lung CT image contained lung lesions, and there were differences between lesion positions and shapes. All samples were divided randomly into training sets and verification sets in 1 : 1 ratio. The training parameter capacity of DPN algorithm model was 5.29 MB. Compared with other algorithms, DPN algorithm model used only a quarter of their parameter capacities (iteration times (epoch), momentum, learning rate, batch size, and weight decay were 400, 0.78, 0.000098, 3.5, and 0.000098, respectively). In addition, the detection accuracy of lung lesions of lung cancer patients reached 88.74%.  Figure 4 demonstrates the detection effect of DPN algorithm model on CT images of lung nodules.

### 3.3. Diagnostic Effects of CT Based on Deep Learning and the Serum Tumor Markers

The patients in the observation group and the control group were compared for four indexes of NSE, CYFRA21, CEA, and SCC. As shown in Figure 5, the observation group had higher NSE, CYFRA21, CEA, and SCC values than the control group, *P* < 0.05.

Subsequently, the patients had the CT examination and serum tumor marker detection. The results showed that the accuracy of CT diagnosis of lung cancer reached 88.37%, the sensitivity was 82.91%, and the specificity was 87.43%, and that the accuracy of serum tumor markers for the diagnosis of lung cancer was 87.34%, the sensitivity was 81.44%, and the specificity was 86.97%. The accuracy of combining CT detection based on deep learning with serum tumor markers was improved to a certain extent, reaching 97.94%, and the sensitivity reached 98.12%, and the specificity was 100%, all of which were higher versus the two methods mentioned before (*P* < 0.05), as shown in Figure 6.

At the same time, the patients were diagnosed by MRI. The diagnosis accuracy rate was 84.38%, the diagnosis sensitivity was 66.66%, and the overall diagnosis specificity was 76.78%. As shown in Figure 7, the accuracy of CT scan based on deep learning for the diagnosis of lung nodules was higher than that of MRI, and the difference was significant (*P* < 0.05).

## 4. Discussion

Based on data analysis, the incidence and mortality of lung diseases, especially lung cancer, have both become clinically nonnegligible key problems. In 2018, the number of dead lung cancer patients accounted for about 18% of total number of deaths worldwide [17, 18]. Compared with that of other diseases, the mortality of lung cancer was higher. Generally, the effective treatment of lung cancer depends on the accurate detection of the disease and the early prevention and treatment. Effective and accurate diagnosis methods can greatly reduce the mortality rate of lung cancer. The current clinical diagnosis of lung cancer can generally be carried out through the following seven techniques, such as chest radiograph (CXR), CT scan, MRI, positron emission tomography (PET), sputum cytology, and breath analysis [19, 20]. All available detection technologies for lung cancer use different markers. These methods have both advantages and limitations. For example, the radiation dose of CXR and CT is low, but MRI and PET have certain limitations in detecting and diagnosing lung nodules [21, 22]. As an important feature of early lung cancer, rapid and effective diagnosis of lung nodules can effectively improve the survival rate of patients with lung diseases.

In addition, lung cancer can also be diagnosed by serum tumor markers combined with imaging methods [23, 24]. Tumor markers refer to substances that are characteristically present in malignant tumor cells or are abnormally produced by malignant tumor cells or produced by the host in response to tumor stimulation, which can reflect the occurrence and development of tumors and monitor the tumor's response to treatment. Tumor markers exist in the tissue, body fluids, and excreta of tumor patients and can be detected by immunological, biological, and chemical methods. In this study, the accuracy of CT diagnosis of lung cancer was 88.37%, the sensitivity was 82.91%, and the specificity was 87.43%. The accuracy of serum tumor markers in the diagnosis of lung cancer was 87.34%, the sensitivity was 81.44%, and the specificity was 86.97%. The accuracy of combining CT based on deep learning and serum tumor markers improved the accuracy to a certain extent, reaching 97.94%, the sensitivity reached 98.12%, and the specificity was 100%.

At present, the most effective technique to detect lung cancer clinically is CT imaging, which can express detailed information about the location and size of lung nodules. In the early stage of cancer, low-dose CT screening can effectively find tumors in the lungs. Compared with traditional radiography technology, it reduces the mortality of patients with lung cancer by 20.0%, and the positive rate of screening has been significantly improved [25]. When the nodules are small, other inspection methods have limitations in diagnosing, while CT can effectively diagnose the patient. Most lung nodules are small in size, about 3 mm in diameter. Radiologists can classify nodules into malignant and benign based on CT. This involves a detailed examination of 3D lung voxels by slicing them into multiple 2D slices [26, 27]. Because CT contains a large amount of information, the analysis must be more precise in order to divide the nodules into malignant and benign. Usually, the possibility of human error in the analysis and diagnosis of CT images will affect detection results of lung nodules [28]. Therefore, the automatic and intelligent diagnosis of lung cancer is important. The model parameter capacity in the training of the DPN algorithm model is 5.29 MB. Compared with other algorithm models, the DPN algorithm model only uses about a quarter of the parameter capacity of them. According to the experimental results, the DPN algorithm model had an accuracy rate of 88.74% for the detection of lung lesions in patients with lung cancer. As an auxiliary method for radiologists, deep learning is used to optimize CT imaging to accurately detect and classify malignant tumors, which is an effective method that has been gradually applied in clinical practice. In addition, Mask-RCNN segmentation algorithm was utilized to segment lung CT images in the research. The results showed that Mask-RCNN segmentation algorithm could not identify the boundaries of images accurately, but it could segment CT images, which was consistent with the results of the study conducted by Zhang et al. [29]. The consistency offered some supports to the results of the research.

## 5. Conclusion

In this study, Mask-RCNN and DPN algorithm were combined to segment CT images of lung cancer patients, and the optimized CT images of pulmonary nodules were analyzed and studied. The results showed that Mask-RCNN combined with DPN algorithm demonstrated better segmentation effects for lung parenchyma CT images than Mask-RCNN or DPN alone, which can effectively improve the diagnostic efficiency of lung cancer CT images, thus improving the diagnostic accuracy and detection efficiency of CT images in lung cancer. However, some limitations in the study should be noted. The sample size is small, which will reduce the power of the study. In the follow-up, an expanded sample size is necessary to strengthen the findings of the study. At present, only automatic detection and labeling of pulmonary nodules can be achieved, but the nature of pulmonary lesions cannot be distinguished, so artificial diagnosis is still needed. In conclusion, the combination of artificial intelligence algorithm and medical imaging technology has broad clinical application prospects and is worthy of clinical promotion.

## Figures and Tables

**Figure 1:** Schematic diagram of segmentation by the Mask-RCNN algorithm.

**Figure 2:** Dual-link structure diagram of the DPN algorithm.

**Figure 3:** The segmentation effect of the Mask-RCNN algorithm on lung CT images.

**Figure 4:** The detection effect of DPN algorithm model on CT images of lung nodules.

**Figure 5:** Diagnostic results of serum tumor markers.

**Figure 6:** Comparison of the diagnostic effects of CT based on deep learning and the serum tumor markers.

**Figure 7:** Comparison of the diagnostic accuracy of CT and MRI on CT images of lung nodules.

## Data Availability

The data used to support the findings of this study are available from the corresponding author upon request.
